# Modeling and Analysis of COVID-19 Spread: The Impacts of Nonpharmaceutical Protocols

**DOI:** 10.1155/2022/7706447

**Published:** 2022-09-02

**Authors:** Reza Shadi, Ahmad Fakharian, Hamid Khaloozadeh

**Affiliations:** ^1^Department of Electrical Engineering, Qazvin Branch, Islamic Azad University, Qazvin, Iran; ^2^Department of Systems and Control Engineering, K.N. Toosi University of Technology, Tehran, Iran

## Abstract

In this study, the extended SEIR dynamical model is formulated to investigate the spread of coronavirus disease (COVID-19) via a special focus on contact with asymptomatic and self-isolated infected individuals. Furthermore, a mathematical analysis of the model, including positivity, boundedness, and local and global stability of the disease-free and endemic equilibrium points in terms of the basic reproduction number, is presented. The sensitivity analysis indicates that reducing the disease contact rate and the transmissibility factor related to asymptomatic individuals, along with increasing the quarantine/self-isolation rate and the contact-tracing process, from the view of flattening the curve for novel coronavirus, are crucial to the reduction in disease-related deaths.

## 1. Introduction

From December 2019 until now, the world is facing a new challenge. The pandemic of COVID-19 was caused by a novel coronavirus and quickly spread to other parts of the world [1]. This severe infectious illness is one of the most contagious viral diseases in humans, and according to statistics, COVID-19 poses a major threat to the health of human society and the economy. The novel coronavirus is transmitted between all age groups of humans through direct close contact with a person while they are infectious, contact with droplets from an infected person's sneeze or cough, touching contaminated objects or surfaces such as cell phones and elevator buttons, and then touching the mouth, nose, and eyes [2]. Coronavirus disease can be transmitted during the asymptomatic incubation phase and for up to two weeks after the onset of symptoms. The World Health Organization (WHO) reported an incubation period for COVID-19 of between 2 and 10 days [3]. Despite the discovery of different platforms of vaccines for the disease, the most effective interventions to break the transmission chain of infection are to maintain physical distance, use face masks, stay away from infected people, identify and quarantine infected people, and stay home. Therefore, people suspected of being infected should be traced and identified immediately and then isolated from others. This means that nonpharmaceutical measures such as physical distancing regulation (stay at least 2 meters away from other people), detecting more cases of COVID-19, effective identification of asymptomatic individuals, self-quarantine, wearing a face mask, and tracing the exposed individuals are still the most effective preventive measures, from the perspective of flattening the curve of COVID-19, to curb the spread of COVID-19 in the suffering community [4–7]. The set of public health strategies that reduce the peak number of people requiring care and mitigate the spread of the disease can be framed in the concept of flattening the curve of the COVID-19 outbreak.

In general, the coronavirus at the onset of the outbreak had devastating effects on all host countries and affected their health and economic infrastructure. COVID-19 has spread to more than 220 countries, and according to the World Health Organization, the virus has affected about 202 million people worldwide, and more than 3.4 million people have died so far [8]. Meanwhile, third-world countries such as Egypt are suffering more irreparable effects. Because of the deficiency of proper infrastructure, the government is not able to impose strict country-wide or regional lockdowns, hospitalize or quarantine all patients, or enforce social distancing regulations. In addition, poor citizens are deprived of government financial support and are therefore forced to carry out daily activities. The first infected case was a Chinese national who was identified at Cairo International Airport and taken to a quarantine center. The first death recorded in Egypt by COVID-19 was on March 20, 2020. Accordingly, the Egyptian government took various preventive measures in March to tackle the effects of the disease, including the closure of educational centers and places of worship. It has also been confirmed as of September 1, 2020, that all travelers intending to travel to this country must provide a polymerase chain reaction (PCR) test certificate for COVID-19 [9].

Mathematical modeling can be applied to a variety of contagious diseases, including Ebola, HIV, influenza, SARS, novel coronavirus epidemics, and heroin, and plays a key role in analyzing epidemiological models, examining the effects of various components, predicting how they will behave, and facilitating disease suppression [10]. Because of the importance of the behavioral pattern of the novel coronavirus, various mathematical models have been developed to investigate the prevalence of the disease. The effect of different control measures as preventive interventions using a new mathematical modeling with quarantine, self-isolation, and public health education and an optimal control approach to determine their contributions to the dynamic transmission of COVID-19 is presented in [4]. The impacts of various preventive control measures on the population dynamics of COVID-19 in Lagos, via an appropriately formulated mathematical model, are carried out in [5]. Kumari et al. [6] applied the SEIAQRDT model, including asymptomatic cases, for the prediction of COVID-19 disease in India. In [7], a deterministic model for the transmission dynamics of the novel coronavirus outbreak incorporating prosocial behavior is provided, wherein the spread of the disease has been studied by unnotified and notified individuals. Mpeshe and Nyerere [11] presented the dynamics of COVID-19 epidemics coupled with fear epidemics. An educational campaign can help reduce fear among people and find possible control mechanisms. Based on the fact that the coronavirus is spread by the travel of people unaware of the disease who are added to the population impulsively, an impulsive epidemic model to indicate the sudden growth in the population is considered in [12]. Zheng et al. [13] considered the role of the diffusion network in the SIR model in order to control and mitigate the COVID-19 outbreak, and the effect of maximum eigenvalue on Turing instability was investigated. In addition, the effect of network parameters on how the disease spreads is examined, and the model stability of the model under the proposed approach is presented via the maximum eigenvalue of the network matrix. Based on real data for Algeria and India, a discrete mathematical model is proposed to provide a simple description of the novel coronavirus spread by Sitthiwirattham et al. [14]. In [15], an optimal analysis of the model for the purpose of assessing the effect of public health education, the effect of personal protective measures, and the effect of treating hospitalized or isolated cases on mitigating transmission of COVID-19 in Ethiopia was conducted. In the absence of pharmaceutical interventions, the immunity system plays a vital role in the recovery of patients. Due to the fact that the immunity system decreases with age, Djilali and Ghanbari [16] proposed the age-structured SEIR model to predict the severity of COVID-19 in South Africa, Brazil, and Turkey. In addition, the effect of isolation on susceptible individuals has been considered, and finally, the end of the disease outbreak in the mentioned countries has been estimated. Given the widespread and rapid prevalence of COVID-19, awareness and prediction of the dynamic behavior of this disease are crucial. Bentout et al. [17] presented an age-structured model for three different countries from three different continents. The proposed model includes hospitalized individuals (via estimating the number of hospital beds required) and the possible infection of the healthcare staff. In addition, the effect of the lack of appropriate personal protective equipment on the spread of the disease is considered. The peak time of the disease and the number of infected people despite medical measures are being studied. The basic reproduction number *ℛ*_0_ as an epidemiological threshold can be examined to characterize the stability of system equilibrium points. In this regard, by examining the existence of the global attractor, two different states for *ℛ*_0_ have been investigated. When *ℛ*_0_ < 1, by using the Fluctuation Lemma, the disease-free equilibrium is globally asymptotically stable. On the other hand, when *ℛ*_0_ > 1, then the system is uniformly persistent [18].

In the event of an epidemic, the effect of unreported individuals on the analysis of disease behavior cannot be ignored. Based on this fact, a mathematical model is presented to investigate the effect of mobility restrictions on active infected individuals in three countries: Algeria, Egypt, and Morocco [19]. The proposed model has been used to estimate the number of unreported patients, people required for hospitalization, and the second wave of outbreaks in the mentioned countries. Shadi et al. [20] proposed an extended SEIR model considering the state of vaccination in order to investigate the effect of pharmaceutical measures in suppressing the progression of novel coronavirus in Iran. Also, to validate the proposed model, it is fitted with the approved daily data reported. A simple analytical expression of the SEIR model has been done by Piovella [21] to investigate the peak number of people in the community and time characteristics affected by the novel coronavirus. Djilali and Bentout [22] presented the SVIR model with weak delay (distributed delay) along with the vaccination state as pharmacological measures to control the spread of the outbreak. In addition, a global compact attractor is determined to investigate the dynamic behavior of the system based on the different numerical values of *ℛ*_0_. Similar to the modeling approach for infection transmission dynamics, this technique can also be applied to modeling drug consumption patterns such as heroin. Like infectious diseases, it is assumed that addiction can be transmitted to nondrug individuals by way of the consumer. The remission of consumption is considered a delay, and the phenomena of Hopf and backward bifurcation have been investigated for the proposed models [23, 24].

In this study, the effects of nonpharmaceutical protocols such as physical distancing regulation, quarantine/self-isolation of patients with clinical symptoms, and tracing of exposed individuals on the spread of COVID-19 using the extended version of the SEIR dynamic model are investigated. In order to evaluate the model, a good fit of the proposed model to the daily confirmed infected cases in Egypt is provided. Other objectives of this paper include investigating the analytical expression and estimating the parameters of the model based on fitted parameters and sensitivity analysis of the basic reproduction number *ℛ*_0_. The rest of this study is organized as follows: The model implementation is presented in Section 2. The basic analysis of the model, including the results of local and global stability of the disease-free and endemic equilibrium points, positivity and boundedness of all trajectories of the proposed model, and the calculation of the basic reproduction number *ℛ*_0_ are examined in Section 3. The model fitting to daily reported cases and estimation of parameters are explained in section 4. Numerical results and discussion are presented in Section 5. Finally, the conclusion is given in Section 6.

## 2. COVID-19 Model Formulation

In this section, the proposed deterministic model, including demographic effects, to study the transmission of the COVID-19 outbreak is presented. To develop the model, the total human population size *N*(*t*) is subdivided into seven epidemiological compartments denoted by susceptible *S*(*t*) (they are not infected yet), exposed *E*(*t*) (they are infected but not yet infectious), asymptomatic infectious *I*_*a*_(*t*) (infectious but undetected), symptomatic infectious *I*_*s*_(*t*) (symptomatic with infectious capacity), quarantined *Q*(*t*), under treatment *H*(*t*) (hospitalized), and recovered *R*(*t*) individuals. The total population at time *t*, denoted by *N*(*t*), is given by *N*(*t*) = *S*(*t*) + *E*(*t*) + *I*_*a*_(*t*) + *I*_*s*_(*t*) + *Q*(*t*) + *H*(*t*) + *R*(*t*). A susceptible person can be infected by direct contact with an infected person from another class. Studies show that asymptomatic patients have a higher viral load than those with symptoms and are capable of transmitting the infection [25, 26]. On the other hand, due to the deficiency of medical infrastructure in Egypt, some people who have a positive PCR test are forced into home quarantine.

Popularly, it is assumed that a self-quarantined person is unable to be a carrier of the disease. However, it is observed that people who are under in-home quarantine and disobey the prevention guidelines are also infected. Practically, family members of these people can also be infected. Let the modification parameter 0 ≤ *ε*_1_ ≤ 1 be considered the effective transmission rate of infection from asymptomatic individuals. Also, the modification parameter 0 ≤ *ε*_2_ ≤ 1 is used for the infection transmission rate owing to self-quarantined COVID-19 patients. After interacting with infected individuals from other groups, a person from the susceptible group can move to the exposed group. The mechanism of how an epidemic is transmitted among all members of a community is expressed by an epidemiological parameter called the force of infection (FOI). According to the aforementioned statements, FOI associated with the model is considered as:

(1) $$\begin{array}{c} \lambda =\frac{\beta \left(I_{s}+\varepsilon_{1}I_{a}+\varepsilon_{2}Q\right)}{N}, \end{array}$$

where the *β* parameter indicates the rate of effective human-to-human contacts that can lead to infection transmission. The parameter *Π* comprises the recruitment rate of the human population per unit value of time, and *μ*_*d*_ is the natural death rate of humans in all classes. The incubation period (the time between exposure to the virus and symptom onset) of COVID-19 disease is 2 days to 2 weeks. After this period, individuals in the exposed compartment become infected at a rate *φ* and, depending on the clinical signs, can move to *I*_*a*_ or *I*_*s*_ classes at *ς* or (1 − *ς*) rates, respectively. In addition, the remaining exposed individuals who have been in contact with infected individuals are identified via the contact-tracing process, and if their test is positive, they join the quarantine compartment at the *ν* rate. The hospitalization rates of symptomatic and quarantined individuals are expressed by *δ* and *q*, respectively. After the infection, the immune system protects the body and mounts a response against that disease [12]. As a result of natural immunity and receiving treatment services in the hospital, symptomatic, asymptomatic, quarantined, and undertreated individuals progress to recover compartments at the rates of *α*, *θ*, *r*, *h*, respectively. Finally, the COVID-19-induced death rate for individuals in the *I*_*s*_, *Q*, and *H* is, respectively, shown by *σ*, *w*, and *ξ*.

Based on the aforementioned statements and descriptions, a flow diagram for the COVID-19 transmission model is illustrated in Figure 1. Consequently, the transmission dynamics of the COVID-19 epidemic is given by a deterministic system of nonlinear differential equations as follows:

(2) $$\begin{array}{c} \begin{array}{c} \frac{\text{d}S}{\text{d}t}=\Pi -\lambda S-\mu_{d}S\\ \frac{\text{d}E}{\text{d}t}=\lambda S-\left(\nu +\varphi +\mu_{d}\right)E\\ \frac{\text{d}I_{a}}{\text{d}t}=\varsigma \varphi E-\left(\alpha +\mu_{d}\right)I_{a}\\ \frac{\text{d}I_{s}}{\text{d}t}=\left(1-\varsigma \right)\varphi E-\left(\theta +\delta +\sigma +\mu_{d}\right)I_{s}\\ \frac{\text{d}Q}{\text{d}t}=\nu E-\left(w+q+r+\mu_{d}\right)Q\\ \frac{\text{d}H}{\text{d}t}=\delta I_{s}+qQ-\left(\xi +h+\mu_{d}\right)H\\ \frac{\text{d}R}{\text{d}t}=\alpha I_{a}+\theta I_{s}+rQ+hH-\mu_{d}R, \end{array} \end{array}$$

with initial conditions *S*_0_ ≥ 0, *E*_0_ ≥ 0, *I*_*a*_0__ ≥ 0, *I*_*s*_0__ ≥ 0, *Q*_0_ ≥ 0, *H*_0_ ≥ 0, and *R*_0_ ≥ 0. It is assumed that all the parameters used in the proposed model are nonnegative, and the biological descriptions related to each one are given in Table 1.

## 3. Basic Analysis of the Model

In this section, some basic analytical outcomes of the COVID-19 model (2), including positivity and boundedness of solution, theoretical presentation of the basic reproduction number *ℛ*_0_ as an epidemiological concept to curb the spread of infectious disease, and stability of disease-free equilibrium (DFE), and endemic equilibrium points in terms of *ℛ*_0_, are provided.

### 3.1. Positivity and Boundedness of the Solution

In order to verify that model (2) is well-posed epidemiologically, it must be shown that all trajectories of the model (2) will remain nonnegative for all *t* > 0 and following nonnegative initial conditions

(3) $$\begin{array}{c} {\left(S\left(0\right),E\left(0\right),I_{a}\left(0\right),I_{s}\left(0\right),Q\left(0\right),H\left(0\right),R\left(0\right)\right)}^{T}\in {\mathbb{R}}_{+}^{7}. \end{array}$$

**Lemma 1 (positivity).**

Assuming that *𝒵*(*t*) = (*S*(*t*), *E*(*t*), *I*_*a*_(*t*), *I*_*s*_(*t*), *Q*(*t*), *H*(*t*), *R*(*t*)) are state variabels of model and *𝒵*(0) ≥ 0 indicates the initial conditions, then all trajectories of the COVID-19 model (2) are nonnegative if they exist for all *t* ≥ 0. Furthermore, lim_*t*⟶∞_sup*N*(*t*) ≤ *Π*/*μ*_*d*_.

**Proof**

Consider *t*_1_ = sup{*t* > 0 : *𝒵*(*t*) > 0 ∈ [0, *t*]}; then multiplying the first equation of the model (2) by the integrating factor exp{*μ*_*d*_*t* + ∫_0_^*t*^*λ*(*τ*)**d***τ*}, we get that

(4) $$\begin{array}{c} \frac{\text{d}}{\text{d}t}\left[S\left(t\right)\exp\left\{\mu_{d}t+\int_{0}^{t}\lambda \left(\tau \right)d\tau \right\}\right]=\Pi \;\exp\left\{\mu_{d}t+\int_{0}^{t}\lambda \left(\tau \right)d\tau \right\}. \end{array}$$

Hence,

(5) $$\begin{array}{c} S\left(t_{1}\right)\;\exp\left\{\mu_{d}t_{1}+\int_{0}^{t_{1}}\lambda \left(\tau \right)d\tau \right\}-S\left(0\right)=\Pi \int_{0}^{t_{1}}\exp\left\{\mu_{d}y+\int_{0}^{y}\lambda \left(\tau \right)d\tau \right\}dy. \end{array}$$

From solving Equation (5), we have

(6) $$\begin{array}{c} S\left(t_{1}\right)=S\left(0\right)\;\exp\left\{-\left(\mu_{d}t_{1}+\int_{0}^{t_{1}}\lambda \left(\tau \right)d\tau \right)\right\}+\exp\left\{-\left(\mu_{d}t_{1}+\int_{0}^{t_{1}}\lambda \left(\tau \right)d\tau \right)\right\}\times \Pi \int_{0}^{t_{1}}\exp\left\{\mu_{d}y+\int_{0}^{y}\lambda \left(\tau \right)d\tau \right\}dy>0. \end{array}$$

Hence, the first equation of model (2) for *t* > 0 is nonnegative. Accordingly, via a similar approach, it can be shown that *𝒵*(0) > 0 for all *t* > 0.

### 3.2. Invariant Region

In the following, the dynamics of the COVID-19 model (2) will be examined in a feasible and closed region with respect to biological considerations:

(7) $$\begin{array}{c} \Omega =\left\{\left(S\left(t\right),E\left(t\right),I_{a}\left(t\right),I_{s}\left(t\right),Q\left(t\right),H\left(t\right),R\left(t\right)\right)\in {\mathbb{R}}_{+}^{7}:0<N\left(t\right)\leq \frac{\Pi }{\mu_{d}}\right\}. \end{array}$$

**Lemma 2 (boundedness).**

The model (2) with nonnegative initial conditions in ℝ_+_^7^ is bounded in the region *Ω*. In other words, the region *Ω* ∈ ℝ_+_^7^ is positively invariant for the COVID-19 model (2) with nonnegative initial conditions in ℝ_+_^7^.

**Proof**

Adding up all the differential equations in the model (2) leads to

(8) $$\begin{array}{c} \frac{\text{d}N\left(t\right)}{\text{d}t}=\Pi -\mu_{d}N\left(t\right)-\sigma I_{s}\left(t\right)-wQ\left(t\right)-\xi H\left(t\right)\leq \Pi -\mu_{d}N\left(t\right). \end{array}$$

It is obvious that d*N*(*t*)/d*t* ≤ 0 if *N*(*t*) ≥ *Π*/*μ*_*d*_.

Using the Grönwall-Bellman inequality and arranging the equation, the solution of (8) is given as follows:

(9) $$\begin{array}{c} \begin{array}{c} N\left(t\right)\leq N\left(0\right)\exp\left(-\mu_{d}t\right)+\frac{\Pi }{\mu_{d}}\left(1-\exp\left(-\mu_{d}t\right)\right). \end{array} \end{array}$$

In particular, if *N*(0) ≤ *Π*/*μ*_*d*_, then it follows from (9) that

(10) $$\begin{array}{c} \begin{array}{cc} N\left(t\right) & \leq \underset{t⟶\infty }{\lim}\sup\;N\left(0\right)\exp\left(-\mu_{d}t\right)+\frac{\Pi }{\mu_{d}}\left(1-\exp\left(-\mu_{d}t\right)\right)=\frac{\Pi }{\mu_{d}}. \end{array} \end{array}$$

Further, if *N*(0) > *Π*/*μ*_*d*_, then *N*(*t*) approaches *Π*/*μ*_*d*_ asymptotically, and the number of infected subpopulations enters *Ω* over time. Therefore, all model solutions are attracted by the region *Ω* eventually.

### 3.3. The Disease-Free Equilibrium State

In epidemiology, a disease-free equilibrium can be established when there is no disease in the community. The proposed model (2) has a disease-free equilibrium *ϵ*_0_, given by

(11) $$\begin{array}{c} \epsilon_{0}=\left(S_{0},0,0,0,0,0,0\right)=\left(\frac{\Pi }{\mu_{d}},0,0,0,0,0,0\right). \end{array}$$

### 3.4. The Basic Reproduction Number *ℛ*_0_

Mathematically, the basic reproduction number is known as a threshold quantity for the stability of the system. In a particular suffering community, the numerical value of *ℛ*_0_ plays a significant role in how to spread the burden of disease. From an epidemiological viewpoint, the reproduction number is defined as the average number of secondary infections when a typical infection enters an entirely susceptible individual [7, 10]. The idea of flattening the curve lies in the basic reproduction number. This means that if *ℛ*_0_ < 1, then the disease can be suppressed and unable to outbreak. However, if *ℛ*_0_ exceeds 1, the disease is an epidemic and can persist. Based on the next-generation operator method [27], by decomposing the RHS of the system (2) corresponding to the infected compartments (i.e., *E*, *I*_*a*_, *I*_*s*_, *Q*, *H*), the relevant matrices to calculate *ℛ*_0_ are given by

(12) $$\begin{array}{c} F=\left(\begin{array}{c} \frac{\beta \left(I_{s}+\varepsilon_{1}I_{a}+\varepsilon_{2}Q\right)S}{N}\\ 0\\ 0\\ 0\\ 0 \end{array}\right),V=\left(\begin{array}{c} k_{1}E\\ k_{2}I_{a}-\varsigma \varphi E\\ k_{3}I_{s}-\left(1-\varsigma \right)\varphi E\\ k_{4}Q-\nu E\\ k_{5}H-\delta I_{s}-qQ \end{array}\right), \end{array}$$

where the nonnegative matrix, *ℱ*, denotes new infection terms, the nonsingular matrix, *𝒱*, represents remaining transfer terms, and

(13) $$\begin{array}{c} k_{1}=\left(\nu +\varphi +\mu_{d}\right), \end{array}$$

(14) $$\begin{array}{c} k_{2}=\left(\alpha +\mu_{d}\right), \end{array}$$

(15) $$\begin{array}{c} k_{3}=\left(\theta +\delta +\sigma +\mu_{d}\right), \end{array}$$

(16) $$\begin{array}{c} k_{4}=\left(w+q+r+\mu_{d}\right), \end{array}$$

(17) $$\begin{array}{c} k_{5}=\left(\xi +h+\mu_{d}\right). \end{array}$$

The Jacobian matrices of *ℱ* and *𝒱* at *ε*_0_ are obtained as follows:

(18) $$\begin{array}{c} F={\left.\left(\frac{\partial F}{\partial \;x_{i}}\right)\right|}_{\epsilon_{0}}=\left(\begin{array}{ccccc} 0 & \beta \varepsilon_{1} & \beta & \beta \varepsilon_{2} & 0\\ 0 & 0 & 0 & 0 & 0\\ 0 & 0 & 0 & 0 & 0\\ 0 & 0 & 0 & 0 & 0\\ 0 & 0 & 0 & 0 & 0 \end{array}\right),\text{and }V={\left.\left(\frac{\partial V}{\partial \;x_{i}}\right)\right|}_{\epsilon_{0}}=\left(\begin{array}{ccccc} k_{1} & 0 & 0 & 0 & 0\\ -\varphi \varsigma & k_{2} & 0 & 0 & 0\\ -\left(1-\varsigma \right)\varphi & 0 & k_{3} & 0 & 0\\ -\nu & 0 & 0 & k_{4} & 0\\ 0 & 0 & -\delta & -q & k_{5} \end{array}\right), \end{array}$$

for *x*_*i*_ = *E*, *I*_*a*_, *I*_*s*_, *Q*, *H*.

Using the definition *ℛ*_0_ = *ρ*(*FV*^−1^), where *ρ* is the spectral radius of *FV*^−1^, the following interpretation is inferred for the basic reproduction number of the proposed model:

(19) $$\begin{array}{c} R_{0}=\frac{\beta \varphi \varsigma \varepsilon_{1}}{k_{1}k_{2}}+\frac{\beta \varphi \left(1-\varsigma \right)}{k_{1}k_{3}}+\frac{\beta \varepsilon_{2}\nu }{k_{1}k_{4}}=R_{I_{a}}+R_{I_{s}}+R_{Q}, \end{array}$$

where *ℛ*_*I*_*a*__, *ℛ*_*I*_*s*__, and *ℛ*_*Q*_ are constituents of *ℛ*_0_ and are contributed by asymptomatic infected individuals, symptomatic infected individuals, and quarantined individuals, respectively.

### 3.5. Stability Analysis of DFE

In this section, we intend to prove the local and global stability of ODE with regard to *ℛ*_0_. Epidemiologically, the meaning of the stability outcome of DFE is that, if *ℛ*_0_ < 1, then a small onset of COVID-19 infections cases will not lead to a COVID-19 persisting in the community. Steady-state analysis has been inspected in the following theorem.

**Theorem 1 .**

The disease-free equilibrium *ϵ*_0_ of the COVID-19 model (2) is locally asymptotically stable (LAS) if and only if *ℛ*_0_ < 1 and unstable if *ℛ*_0_ > 1.

The Jacobian matrix corresponding to the system (2) at the *ε*_0_ is as follows:

(20) $$\begin{array}{c} J\left(\varepsilon_{0}\right)=\left(\begin{array}{ccccccc} -\mu_{d} & 0 & -\beta \varepsilon_{1} & -\beta & -\beta \varepsilon_{2} & 0 & 0\\ 0 & -k_{1} & \beta \varepsilon_{1} & \beta & \beta \varepsilon_{2} & 0 & 0\\ 0 & \varsigma \varphi & -k_{2} & 0 & 0 & 0 & 0\\ 0 & \left(1-\varsigma \right)\varphi & 0 & -k_{3} & 0 & 0 & 0\\ 0 & \nu & 0 & 0 & -k_{4} & 0 & 0\\ 0 & 0 & 0 & \delta & q & -k_{5} & 0\\ 0 & 0 & \alpha & \theta & r & h & -\mu_{d} \end{array}\right). \end{array}$$

It is clear that *s*_1_ = *s*_2_ = −*μ*_*d*_, *s*_3_ = −*k*_5_ have negative real parts. The remaining eigenvalues (four) can be obtained through the roots of the following characteristic equation:

(21) $$\begin{array}{c} \Delta \left(s\right)=s^{4}+a_{3}s^{3}+a_{2}s^{2}+a_{1}s+a_{0}=0, \end{array}$$

where

(22) $$\begin{array}{c} a_{3}=k_{1}+k_{2}+k_{3}+k_{4}, \end{array}$$

(23) $$\begin{array}{c} a_{2}=k_{1}k_{2}\left(1-R_{I_{a}}\right)+k_{1}k_{3}\left(1-R_{I_{s}}\right)+k_{1}k_{4}\left(1-R_{Q}\right)+k_{2}k_{3}+k_{2}k_{4}+k_{3}k_{4}, \end{array}$$

(24) $$\begin{array}{c} a_{1}=k_{1}k_{2}k_{3}\left(1-R_{I_{a}}-R_{I_{s}}\right)+k_{1}k_{2}k_{4}\left(1-R_{Q}-R_{I_{a}}\right)+k_{1}k_{3}k_{4}\left(1-R_{Q}-R_{I_{s}}\right)+k_{2}k_{3}k_{4}, \end{array}$$

(25) $$\begin{array}{c} a_{0}=k_{1}k_{2}k_{3}k_{4}\left(1-R_{0}\right). \end{array}$$

Since *ℛ*_*I*_*a*__, *ℛ*_*I*_*s*__, and *ℛ*_*Q*_ are all positive and *ℛ*_0_ = *ℛ*_*I*_*a*__ + *ℛ*_*I*_*s*__ + *ℛ*_*Q*_, it is obvious that the coefficients *a*_*i*_ for *i* = 0, 1, 2, 3 are positive and the last statement is positive whenever *ℛ*_0_ < 1. Furthermore, the Routh-Hurwitz stability criterion can be used to ensure the stability of model (2) at the DFE. Since all the parameters of the proposed model are positive, it can be easily seen that, if *ℛ*_0_ < 1, then the Routh-Hurwitz conditions are met, *a*_0_ > 0, *a*_0_*a*_1_ − *a*_2_ > 0, (*a*_0_*a*_1_ − *a*_2_)*a*_2_ − *a*_0_^2^*a*_3_ > 0, and *a*_3_ > 0. Accordingly, the DFE *ε*_0_ is locally asymptotically stable if *ℛ*_0_ < 1.

To show that the mitigate of the COVID-19 pandemic is independent of the initial number of infected cases in a particular community, it must be demonstrated that the disease-free equilibrium is globally asymptotically stable (GAS), if *ℛ*_0_ < 1.

**Theorem 2 .**

The DFE *ϵ*_0_ is globally asymptotically stable for the model (2), if *ℛ*_0_ < 1.

**Proof**

Consider the following Lyapunov function candidate for the COVID-19 model (2) defined by

(26) $$\begin{array}{c} Y\left(t\right)=A_{1}E\left(t\right)+A_{2}I_{a}\left(t\right)+A_{3}I_{s}\left(t\right)+A_{4}Q\left(t\right), \end{array}$$

where *A*_*i*_, *i* = 1, 2, 3, 4, are positive coefficients that are determined later.

Making the time derivative of (26) and substituting the expressions from system (2), into the Lyapunov derivative $\dot{Y}\left(t\right)$, we have

(27) $$\begin{array}{c} \frac{\text{dY}\left(t\right)}{\text{d}t}=A_{1}\dot{E}\left(t\right)+A_{2}{\dot{I}}_{a}\left(t\right)+A_{3}{\dot{I}}_{s}\left(t\right)+A_{4}\dot{Q}\left(t\right)=A_{1}\left[\left(\frac{\beta \left(I_{s}+\varepsilon_{1}I_{a}+\varepsilon_{2}Q\right)}{N}\right)S-k_{1}E\right]+A_{2}\left[\varsigma \varphi E-k_{2}I_{a}\right]+A_{3}\left[\left(1-\varsigma \right)\varphi E-k_{3}I_{s}\right]+A_{4}\left[\nu E-k_{4}Q\right];\left(Since\;N\geq S\right),\leq A_{1}\left[\left(\beta \left(I_{s}+\varepsilon_{1}I_{a}+\varepsilon_{2}Q\right.\right)-k_{1}E\right]+A_{2}\left[\varsigma \varphi E-k_{2}I_{a}\right]+A_{3}\left[\left(1-\varsigma \right)\varphi E-k_{3}I_{s}\right]+A_{4}\left[\nu E-k_{4}Q\right]=\left[A_{2}\varsigma \varphi +A_{3}\left(1-\varsigma \right)\varphi +A_{4}\nu -A_{1}k_{1}\right]E+\left[A_{1}\beta \varepsilon_{1}-A_{2}k_{2}\right]I_{a}+\left[A_{1}\beta -A_{3}k_{3}\right]I_{s}+\left[A_{1}\beta \varepsilon_{2}-A_{4}k_{4}\right]Q=A_{1}k_{1}\left[\frac{A_{2}\varsigma \varphi }{A_{1}k_{1}}+\frac{A_{3}\left(1-\varsigma \right)\varphi }{A_{1}k_{1}}+\frac{A_{4}\nu }{A_{1}k_{1}}-1\right]E+\left[A_{1}\beta \varepsilon_{1}-A_{2}k_{2}\right]I_{a}+\left[A_{1}\beta -A_{3}k_{3}\right]I_{s}+\left[A_{1}\beta \varepsilon_{2}-A_{4}k_{4}\right]Q. \end{array}$$

Now choosing *A*_1_ = 1, *A*_2_ = *βε*_1_/*k*_2_, *A*_3_ = *β*/*k*_3_, and *A*_4_ = *βε*_2_/*k*_4_ and carrying out some algebraic manipulations and simplifications, we obtained

(28) $$\begin{array}{c} \frac{\text{dY}\left(t\right)}{\text{d}t}\leq k_{1}\left(R_{0}-1\right)E. \end{array}$$

It results that, if *ℛ*_0_ < 1, then dY(*t*)/d*t* ≤ 0. Further, with equality dY(*t*)/d*t* = 0, if and only if *E* = 0, *I*_*a*_ = 0, *I*_*s*_ = 0, and *Q* = 0. Eventually, due to the LaSalle's Invariance Principle [28], it can be concluded that the largest compact invariant set in *Ω* is the singleton set *ε*_0_. According to this, *ε*_0_ is globally asymptotically stable in *Ω*. The result of this theory will be depicted graphically.

### 3.6. Existence of Endemic Equilibrium Point

In this subsection, the existence of the endemic equilibrium point (EEP) is examined.

**Lemma 3 .**

Let *Π* = *μ*_*d*_*N*. For the proposed model (2), there is a positive endemic equilibrium point if *ℛ*_0_ > 1.

**Proof**

The EEP of the proposed model at *ε*_*EEP*_ = (*S*^∗^, *E*^∗^, *I*_*a*_^∗^, *I*_*s*_^∗^, *Q*^∗^, *H*^∗^, *R*^∗^) is obtained by equalizing the right-hand side of model (2) with zero; hence

(29) $$\begin{array}{c} \left\{\begin{array}{c} S^{*}=\frac{N}{R_{0}},\\ E^{*}=\frac{\mu_{d}N\left(R_{0}-1\right)}{R_{0}\left(\nu +\varphi +\mu_{d}\right)},\\ I_{a}^{*}=\frac{\varsigma \varphi \mu_{d}N\left(R_{0}-1\right)}{R_{0}\left\{\left(\nu +\varphi +\mu_{d}\right)\left(\alpha +\mu_{d}\right)\right\}},\\ I_{s}^{*}=\frac{\left(1-\varsigma \right)\varphi \mu_{d}N\left(R_{0}-1\right)}{R_{0}\left\{\left(\nu +\varphi +\mu_{d}\right)\left(\theta +\delta +\sigma +\mu_{d}\right)\right\}},\\ Q^{*}=\frac{\nu \mu_{d}N\left(R_{0}-1\right)}{R_{0}\left\{\left(\nu +\varphi +\mu_{d}\right)\left(w+q+r+\mu_{d}\right)\right\}},\\ H^{*}=\frac{\delta \left(1-\varsigma \right)\varphi \mu_{d}N\left(R_{0}-1\right)}{R_{0}\left\{\left(\nu +\varphi +\mu_{d}\right)\left(\theta +\delta +\sigma +\mu_{d}\right)\left(\xi +h+\mu_{d}\right)\right\}}\\ +\frac{q\nu \mu_{d}N\left(R_{0}-1\right)}{R_{0}\left\{\left(\nu +\varphi +\mu_{d}\right)\left(w+q+r+\mu_{d}\right)\left(\xi +h+\mu_{d}\right)\right\}},\\ R^{*}=\frac{\alpha I_{a}^{*}+\theta I_{s}^{*}+rQ^{*}+hH^{*}}{\mu_{d}}. \end{array}\right. \end{array}$$

It can be seen that a positive EEP exists for *ℛ*_0_ > 1. Hence, model (2) has an endemic equilibrium point if and only if *ℛ*_0_ exceeds 1.

### 3.7. Local Stability of Endemic Equilibrium Point

The local stability analysis of EEP is investigated by the following statement:

**Theorem 3 .**

The EEP of the proposed model (2) at *ϵ*_*EEP*_ is locally asymptotically stable, when *ℛ*_0_ > 1.

**Proof**

The Jacobian matrix corresponding to the model (2) at endemic equilibrium point *ε*_*EEP*_ is obtained as follows:

(30) $$\begin{array}{c} J\left(\varepsilon_{EEP}\right)=\left(\begin{array}{ccccccc} -k_{6}-\mu_{d} & 0 & -\varepsilon_{1}k_{7} & -k_{7} & -\varepsilon_{2}k_{7} & 0 & 0\\ k_{6} & -k_{1} & \varepsilon_{1}k_{7} & k_{7} & \varepsilon_{2}k_{7} & 0 & 0\\ 0 & \varsigma \varphi & -k_{2} & 0 & 0 & 0 & 0\\ 0 & \left(1-\varsigma \right)\varphi & 0 & -k_{3} & 0 & 0 & 0\\ 0 & \nu & 0 & 0 & -k_{4} & 0 & 0\\ 0 & 0 & 0 & \delta & q & -k_{5} & 0\\ 0 & 0 & \alpha & \theta & r & h & -\mu_{d} \end{array}\right), \end{array}$$

where *k*_6_ = *β*(*I*_*s*_^∗^ + *ε*_1_*I*_*a*_^∗^ + *ε*_2_*Q*^∗^)/*N* and *k*_7_ = *β*(*S*^∗^/*N*).

In the aforementioned Jacobian matrix, the two eigenvalues *e*_1_ = −*μ*_*d*_, *e*_2_ = −*k*_5_ have the negative sign of the real part. The sign of the other eigenvalues is determined by characteristic polynomial (31) as follows:

(31) $$\begin{array}{c} \Delta \left(e\right)=e^{5}+b_{4}e^{4}+b_{3}e^{3}+b_{2}e^{2}+b_{1}e+b_{0}=0, \end{array}$$

where the coefficients *b*_*i*_, *i* = 0, ⋯, 4, are positive and given by

(32) $$\begin{array}{c} b_{4}=k_{1}+k_{2}+k_{3}+k_{4}+k_{6}+\mu_{d}>0,\\ b_{3}=\frac{k_{1}k_{2}\left(R_{I_{s}}+R_{Q}\right)+k_{1}k_{3}\left(R_{I_{a}}+R_{Q}\right)+k_{1}k_{4}\left(R_{I_{a}}+R_{I_{s}}\right)}{R_{0}}+k_{2}k_{3}+k_{2}k_{4}+k_{3}k_{4}+k_{1}k_{6}+k_{2}k_{6}+k_{3}k_{6}+k_{4}k_{6}+k_{1}\mu_{d}+k_{2}\mu_{d}+k_{3}\mu_{d}+k_{4}\mu_{d}>0,\\ b_{2}=k_{1}k_{2}k_{3}\left(\frac{R_{Q}}{R_{0}}\right)+k_{1}k_{2}k_{4}\left(\frac{R_{I_{s}}}{R_{0}}\right)+k_{1}k_{3}k_{4}\left(\frac{R_{I_{a}}}{R_{0}}\right)+\frac{k_{1}k_{2}\mu_{d}\left(R_{I_{s}}+R_{Q}\right)+k_{1}k_{3}\mu_{d}\left(R_{I_{a}}+R_{Q}\right)+k_{1}k_{4}\mu_{d}\left(R_{I_{a}}+R_{I_{s}}\right)}{R_{0}}+k_{1}k_{2}k_{6}+k_{2}k_{3}k_{4}+k_{1}k_{3}k_{6}+k_{1}k_{4}k_{6}+k_{2}k_{3}k_{6}+k_{2}k_{4}k_{6}+k_{3}k_{4}k_{6}+k_{2}k_{3}\mu_{d}+k_{2}k_{4}\mu_{d}+k_{3}k_{4}\mu_{d}>0,\\ b_{1}=k_{1}k_{2}k_{3}\mu_{d}\left(\frac{R_{Q}}{R_{0}}\right)+k_{1}k_{2}k_{4}\mu_{d}\left(\frac{R_{I_{s}}}{R_{0}}\right)+k_{1}k_{3}k_{4}\mu_{d}\left(\frac{R_{I_{a}}}{R_{0}}\right)+k_{1}k_{2}k_{3}k_{6}+k_{1}k_{2}k_{4}k_{6}+k_{1}k_{3}k_{4}k_{6}+k_{2}k_{3}k_{4}k_{6}+k_{2}k_{3}k_{4}\mu_{d}>0,\\ b_{0}=k_{1}k_{2}k_{3}k_{4}k_{6}>0. \end{array}$$

Based on (19) and fulfilling the Routh-Hurwitz stability criteria, all eigenvalues of the characteristic Equation (31) have a negative real part, and the EEP of the proposed model (2) is locally asymptotically stable if *ℛ*_0_ > 1.

### 3.8. Global Stability of Endemic Equilibrium Point

The following statement implies the global stability analysis of the endemic equilibrium point:

**Theorem 4 .**

The EEP of the proposed model (2) is globally asymptotically stable in the region *Ω*, if *ℛ*_0_ > 1.

**Proof**

In this regard, consider the following Lyapunov function:

(33) $$\begin{array}{c} \Gamma \left(S,E,I_{a},I_{s},Q,H,R\right)=\left(S-S^{*}-S^{*}\ln\frac{S}{S^{*}}\right)+\left(E-E^{*}-E^{*}\ln\frac{E}{E^{*}}\right)+\left(I_{a}-I_{a}^{*}-I_{a}^{*}\ln\frac{I_{a}}{I_{a}^{*}}\right)+\left(I_{s}-I_{s}^{*}-I_{s}^{*}\ln\frac{I_{s}}{I_{s}^{*}}\right)+\left(Q-Q^{*}-Q^{*}\ln\frac{Q}{Q^{*}}\right)+\left(H-H^{*}-H^{*}\ln\frac{H}{H^{*}}\right)+\left(R-R^{*}-R^{*}\ln\frac{R}{R^{*}}\right). \end{array}$$

Taking the time derivative of (33) with respect to time and replacing the expressions of model (2) lead to

(34) $$\begin{array}{c} \frac{d\Gamma }{\text{d}t}=\left(\frac{S-S^{*}}{S}\right)\dot{S}+\left(\frac{E-E^{*}}{E}\right)\dot{E}+\left(\frac{I_{a}-I_{a}^{*}}{I_{a}}\right){\dot{I}}_{a}+\left(\frac{I_{s}-I_{s}^{*}}{I_{s}}\right){\dot{I}}_{s}+\left(\frac{Q-Q^{*}}{Q}\right)\dot{Q}+\left(\frac{H-H^{*}}{H}\right)\dot{H}+\left(\frac{R-R^{*}}{R}\right)\dot{R}=\left(1-\frac{S^{*}}{S}\right)\left(\Pi -\frac{\beta \left(I_{s}+\varepsilon_{1}I_{a}+\varepsilon_{2}Q\right)\left(S-S^{*}\right)}{N}-\mu_{d}\left(S-S^{*}\right)-\left(\frac{\beta \left(I_{s}+\varepsilon_{1}I_{a}+\varepsilon_{2}Q\right)S^{*}}{N}+\mu_{d}S^{*}\right)\right)+\left(1-\frac{E^{*}}{E}\right)\left(\frac{\beta \left(I_{s}+\varepsilon_{1}I_{a}+\varepsilon_{2}Q\right)S}{N}-\left(\nu +\varphi +\mu_{d}\right)\left(E-E^{*}\right)-\left(\nu +\varphi +\mu_{d}\right)E^{*}\right)+\left(1-\frac{I_{a}^{*}}{I_{a}}\right)\left(\varsigma \varphi E-\left(\alpha +\mu_{d}\right)\left(I_{a}-I_{a}^{*}\right)-\left(\alpha +\mu_{d}\right)I_{a}^{*}\right)+\left(1-\frac{I_{s}^{*}}{I_{s}}\right)\left(\left(1-\varsigma \right)\varphi E-\left(\theta +\delta +\sigma +\mu_{d}\right)\left(I_{s}-I_{s}^{*}\right)-\left(\theta +\delta +\sigma +\mu_{d}\right)I_{s}^{*}\right)+\left(1-\frac{Q*}{Q}\right)\left(\nu E-\left(w+q+r+\mu_{d}\right)\left(Q-Q^{*}\right)-\left(w+q+r+\mu_{d}\right)Q^{*}\right)+\left(1-\frac{H*}{H}\right)\left(\delta I_{s}+qQ-\left(\xi +h+\mu_{d}\right)\left(H-H^{*}\right)-\left(\xi +h+\mu_{d}\right)H^{*}\right)+\left(1-\frac{R*}{R}\right)\left(\alpha I_{a}+\theta I_{s}+rQ+hH-\mu_{d}\left(R-R^{*}\right)-\mu_{d}R^{*}\right). \end{array}$$

By manipulating and rearranging terms, we obtain

(35) $$\begin{array}{c} \frac{d\Gamma }{\text{d}t}=\Pi -\left(\frac{S^{*}}{S}\Pi +S^{*}\lambda +S^{*}\mu_{d}\right)+\frac{{S^{*}}^{2}}{S}\left(\lambda +\mu_{d}\right)-\frac{{\left(S-S^{*}\right)}^{2}}{S}\left(\lambda +\mu_{d}\right)+\lambda S-\frac{E^{*}}{E}\lambda S-k_{1}E^{*}+\frac{{E^{*}}^{2}}{E}k_{1}-\frac{{\left(E-E^{*}\right)}^{2}}{E}k_{1}+\varsigma \varphi E-\frac{I_{a}^{*}}{I_{a}}\varsigma \varphi E-k_{2}I_{a}^{*}+\frac{{I_{a}^{*}}^{2}}{I_{a}}k_{2}-\frac{{\left(I_{a}-I_{a}^{*}\right)}^{2}}{I_{a}}k_{2}+\left(1-\varsigma \right)\varphi E-\frac{I_{s}^{*}}{I_{s}}\left(1-\varsigma \right)\varphi E-k_{3}I_{s}^{*}+\frac{{I_{s}^{*}}^{2}}{I_{s}}k_{3}-\frac{{\left(I_{s}-I_{s}^{*}\right)}^{2}}{I_{s}}k_{3}+\nu E-\frac{Q^{*}}{Q}\nu E-k_{4}Q^{*}+\frac{{Q^{*}}^{2}}{Q}k_{4}-\frac{{\left(Q-Q^{*}\right)}^{2}}{Q}k_{4}+\left(\delta I_{s}+qQ\right)-\frac{H^{*}}{H}\left(\delta I_{s}+qQ\right)-k_{5}H^{*}+\frac{{H^{*}}^{2}}{H}k_{5}-\frac{{\left(H-H^{*}\right)}^{2}}{H}k_{5}+\left(\alpha I_{a}+\theta I_{s}+rQ+hH\right)-\frac{R^{*}}{R}\left(\alpha I_{a}+\theta I_{s}+rQ+hH\right)-\mu_{d}R^{*}+\frac{{R^{*}}^{2}}{R}\mu_{d}-\frac{{\left(R-R^{*}\right)}^{2}}{R}\mu_{d}. \end{array}$$

Next, we can write *d*Γ/d*t* = *χ*_1_ − *χ*_2_, where

(36) $$\begin{array}{c} \chi_{1}=\Pi +\frac{{S^{*}}^{2}}{S}\left(\lambda +\mu_{d}\right)+\lambda S+\frac{{E^{*}}^{2}}{E}k_{1}+\varsigma \varphi E+\frac{{I_{a}^{*}}^{2}}{I_{a}}k_{2}+\left(1-\varsigma \right)\varphi E+\frac{{I_{s}^{*}}^{2}}{I_{s}}k_{3}+\nu E+\frac{{Q^{*}}^{2}}{Q}k_{4}+\left(\delta I_{s}+qQ\right)+\frac{{H^{*}}^{2}}{H}k_{5}+\left(\alpha I_{a}+\theta I_{s}+rQ+hH\right)+\frac{{R^{*}}^{2}}{R}\mu_{d},\\ \chi_{2}=\left(\frac{S^{*}}{S}\Pi +S^{*}\lambda +S^{*}\mu_{d}\right)+\frac{{\left(S-S^{*}\right)}^{2}}{S}\left(\lambda +\mu_{d}\right)+\frac{E^{*}}{E}\lambda S+k_{1}E^{*}+\frac{{\left(E-E^{*}\right)}^{2}}{E}k_{1}+\frac{I_{a}^{*}}{I_{a}}\varsigma \varphi E+k_{2}I_{a}^{*}+\frac{{\left(I_{a}-I_{a}^{*}\right)}^{2}}{I_{a}}k_{2}+\frac{I_{s}^{*}}{I_{s}}\left(1-\varsigma \right)\varphi E+k_{3}I_{s}^{*}+\frac{{\left(I_{s}-I_{s}^{*}\right)}^{2}}{I_{s}}k_{3}+\frac{Q^{*}}{Q}\nu E+k_{4}Q^{*}+\frac{{\left(Q-Q^{*}\right)}^{2}}{Q}k_{4}+\frac{H^{*}}{H}\left(\delta I_{s}+qQ\right)+k_{5}H^{*}+\frac{{\left(H-H^{*}\right)}^{2}}{H}k_{5}+\frac{R^{*}}{R}\left(\alpha I_{a}+\theta I_{s}+rQ+hH\right)+\mu_{d}R^{*}+\frac{{\left(R-R^{*}\right)}^{2}}{R}\mu_{d}. \end{array}$$

Since it is assumed that all parameters of model (2) are nonnegative, we have *d*Γ/d*t* ≤ 0 for *χ*_1_ ≤ *χ*_2_. Furthermore, when *χ*_1_ = *χ*_2_, then *d*Γ/d*t* = 0. In other words, if *t*⟶∞, it can be stated that (*S*, *E*, *I*_*a*_, *I*_*s*_, *Q*, *H*, *R*)⟶(*S*^∗^, *E*^∗^, *I*_*a*_^∗^, *I*_*s*_^∗^, *Q*^∗^, *H*^∗^, *R*^∗^). Finally, by using LaSalle's Invariance Principle [28], the EEP of the proposed model is globally asymptotically stable.

Theory 7 states that without considering the number of infected people at the onset, when *ℛ*_0_ > 1, the virus will persist and spread widely in the community.

### 3.9. Sensitivity Analysis and Discussion

In this part, the relative contribution of model parameters to how the disease persists in the population is investigated. Sensitivity analysis leads to clear insights for a precise focus on targeted preventive interventions (pharmacological treatments and nonpharmaceutical protocols) to control the prevalence of disease transmission in order to reduce disease-induced deaths.

In order to evaluate the efficacy of model parameters in preventive and therapeutic strategies, the normalized forward sensitivity index of basic reproduction number can be performed to measure the relative changes of *ℛ*_0_ with respect to the vital parameters of the model [29, 30].

**Definition 1 .**

The normalized forward sensitivity index of *ℛ*_0_, which depends differentiably on the parameter Θ, is defined by

(37) $$\begin{array}{c} S_{\Theta }^{R_{0}}≔\frac{\Theta }{R_{0}}\times \frac{\partial R_{0}}{\partial \Theta }. \end{array}$$

In (37), if the sign of the sensitivity index is positive for a parameter, the rate of infection transmission grows with the relevant parameter. The index with a higher magnitude can be considered a controlling factor in disease transmission. It should be noted that some parameters are beyond human control and cannot be considered measures to control disease transmission, such as the death rate and population growth rate.

The sign of the calculated sensitivity indices of *ℛ*_0_ with respect to some parameters of model (2), using the formula given in (37), is tabulated in Table 2. Our findings show that the parameters *β*, *ε*_1_, *ε*_2_, and *ς* have a positive sign, implying that the value of *ℛ*_0_ will increase as these parameters are increased. While the remaining parameters have a negative sign, it means that the value of *ℛ*_0_ will decrease for higher values of these parameters.

## 4. Parameter Estimation and Model Validation

The model validation process determines how accurate a mathematical model is in representing real data. Due to the fact that many aspects of the onset of the novel coronavirus are still unknown, the parameter estimation process has an effective contribution to forecasting the dynamical behavior of the COVID-19 pandemic. In this section, the data fitting using model (2) to the confirmed COVID-19-infected cases in Egypt is investigated. In order to achieve a better fit of the model solution to the actual data, the biological parameters of the model are estimated via a nonlinear least-square fitting approach. To do this, we consider the daily cumulative number of reported cases from February 14, 2020, to May 23, 2020, reported in Egypt. The confirmed reported data was obtained from [31].

For the proposed model, the demographic parameters can be estimated, for example, the natural death rate *μ*_*d*_ for an Egyptian citizen is 1/72.54 per year (3.777 × 10^−5^ per day) according to the WHO report (year 2020). The total population of Egypt in 2020 is *N*(0) = 102,334,404 [32]. In this study, we assume that the population size is nonconstant, and thus, the birth rate is estimated to be *Π* = *N*(0) × *μ*_*d*_ ≈ 3865.

The nonlinear differential equations of model (2) can be exhaustively deemed to be as follows:

(38) $$\begin{array}{c} \frac{\text{d}Z}{\text{d}t}=G\left(t,Z,\Phi \right),Z\left(t_{0}\right)=Z_{0}, \end{array}$$

where *𝒢* is a time-dependent function, *𝒵* is the vector of state variables, and *Φ* is a set of model parameters to be estimated.

In this study, during the specified time period, the nonlinear differential equations of model (2) are solved numerically via the ode45 package, and the resulting solutions are used to determine the best fit of the model parameters using an optimal estimation lsqcurvefit routine with the trust-region-reflective algorithm in the MATLAB© software [15, 30, 33]. This approach minimizes the sum of the squared residuals:

(39) $$\begin{array}{c} \hat{\Phi }=\overset{n}{\underset{i=1}{\sum }}{\left(y_{t_{i}}-{\tilde{y}}_{t_{i}}\right)}^{2}, \end{array}$$

where *n* denotes the total number of available actual data points for the fitting process. In the objective function (39), *y*_*t*_*i*__ is the confirmed reported data, and ${\tilde{y}}_{t_{i}}$ is the solution of the model associated with the model parameters *Φ*. Accordingly, to obtain the best-fit model parameters, the following objective function should be minimized:

(40) $$\begin{array}{c} \left\{\begin{array}{cc} \min & \hat{\Phi }\\ subject\;to & \left(38\right). \end{array}\right. \end{array}$$

The model fitting with daily confirmed reported cases is illustrated in Figure 2. It can be seen that the model fitting is good for the real data. The estimated parameters for COVID-19 disease in Egypt are given in Table 3. Taking into account the estimated parameters, the approximate value of the basic reproduction number for Egypt is *ℛ*_0_ ≈ 2.6408. Also, the two metrics for evaluating the accuracy of the model fitting process are considered: mean absolute error (MAE) and root mean squared error (RMSE). For model fitting of Egypt, the values obtained are *RMSE* = 54.64 and *MAE* = 290.92. Accordingly, the numerical values obtained for the two relevant indicators demonstrate that the data fitting process is quite good.

In the following, some numerical simulations are investigated in order to validate the model and evaluate the effect of some nonpharmaceutical protocol parameters on the persistence or eradication of the infectious COVID-19 communicable disease.  Figure 3 shows the estimated number of symptomatic COVID-19 cases with the daily confirmed reported data in Egypt. Using the numerical values of fixed parameters from Table 3, the sensitivity indices for model (2) are depicted in Figure 4. It can be observed that the parameter *β* has the highest sensitivity value with a high positive influence compared to all other parameters. This means that an alteration of 1% (increase or decrease) in the value of parameter *β* will lead to a variation (increase or decrease) of the *ℛ*_0_ by 1%.

## 5. Numerical Results and Discussion

In order to perform numerical simulations, we consider the total population of Egypt in 2020 as *N*(0) = 102,334,404. Furthermore, at the onset of the COVID-19 outbreak, the initial populations of exposed and asymptomatic individuals were assumed to be *E*(0) = 500 and *I*_*a*_(0) = 150, respectively. The initial symptomatic infected population as given in the confirmed data is *I*_*s*_(0) = 1. It should be noted that there were no treated, self-quarantined, and recovered individuals initially, so *H*(0) = 0, *Q*(0) = 0, and *R*(0) = 0, respectively. Hence, the initial size of the susceptible population is given as *S*(0) = *N*(0) − *E*(0) − *I*_*a*_(0) − *I*_*s*_(0) − *Q*(0) − *H*(0) − *R*(0).

In order to investigate the effect of the contact rate *β* on the burden of the COVID-19 communicable epidemic, various numerical values of this parameter have been considered. The dynamic behavior of the infectious population due to an increase in physical distancing (reduction in *β*) is shown in Figure 5. Clearly, by decreasing the disease contact rate from baseline social distancing (keeping a distance of at least 2 meters away from others) to strict social distancing regulation at least a 40% reduction in *β* (staying at home or, more preferably, lockdown), the total number of COVID-19 infective individuals will decrease substantially. Accordingly, in the first stage of applying preventive policies and preventive interventions, the Egyptian government must eliminate effective contact rates and comply with social distancing regulations during the COVID-19 crisis as far as possible.

The novel coronavirus can be transmitted by people who are infected but never have clinical characteristics (or who experience very mild or almost unrecognizable symptoms). Undoubtedly, these people have a significant role in contributing to the disease burden without their own knowledge. Asymptomatic carriers are an important source of infection, and they are known as silent carriers. The effect of *ε*_1_ parameter is depicted in Figure 6. The total number of infected individuals decreases when *ε*_1_ decreases. On the other hand, the effect of *ε*_2_ parameter on how infection is transmitted from quarantined/self-isolated patients is illustrated in Figure 7. It is observed that reducing this parameter does not have much effect on the epidemic's burden. Obviously, those COVID-19 patients who are in compulsory quarantine or self-isolation are separated from other people, and no one is allowed to meet them. Therefore, this class of infected people does not help to curtail the burden of the disease as long as they are in compulsory quarantine and home isolation.

In the fight against the novel coronavirus, contact tracing is regarded as critical in attempting to prevent the onset of an outbreak. When a patient with suspected COVID-19 is identified, the patient should be immediately isolated from the rest of the population.  Figure 8 states that identifying exposed individuals and strictly enforcing the contact tracking policy can reduce further transmission dramatically. In Figure 9, the effects of the hospitalization rate of symptomatic individuals at different values are illustrated. It is projected that an increase in the hospitalization rate of people with clinical signs and symptoms has no significant effect on the disease burden.

According to the results, the impact of *ε*_2_ parameter is not as effective as taking efforts to curb disease contact rates among infectious (*β*) and asymptomatic (*ε*_1_) ones. Since, in the case of the novel coronavirus, a large fraction of transmission occurs before the onset of clinical symptoms, a mandatory quarantine or stringent contact-tracing measure (*ν*) to identify exposed people will be required to tackle the disease burden in Egypt.

It should be noted that *ℛ*_0_ is not a fixed number in general, and the basic reproductive number is a function of some biological parameters. Hence, the behavior of *ℛ*_0_ according to variations of two arbitrary parameters simultaneously can be depicted in contour plots (Figures 10–13).  Figure 10 represents an increase in *ℛ*_0_ with increasing effective rates for both asymptomatic and quarantined individuals. It implies that, to make sure *ℛ*_0_ < 1, reducing the values of the effective contact rates *ε*_1_ and *ε*_2_ must be strictly considered in the suffering community. It is clear from Figure 11 that reducing the incubation period of the new coronavirus, while improving the hospitalization rate of symptomatic people, can reduce the *ℛ*_0_ value below 1. According to the results obtained from Figures 12 and 13, it can be said that compliance with social distancing (reduction of effective contact rate *β*) by about 40%, along with increasing preventive measures such as contact-tracing process and self-quarantine at home for exposed individuals (*ν*) as well as an increased hospitalization rate (*δ*), can mitigate the burden of the epidemic.

In order to graphically evaluate the global stability of the COVID-19 transmission model (2), we examine the convergence of model trajectories at disease-free equilibrium regardless of the initial condition of the infected individuals. The results in Figure 14 confirm the predefined Theorem 4.

## 6. Conclusion

In this study, a deterministic mathematical model has been presented to analyze the dynamical behavior of the COVID-19 epidemic in Egypt, and it has been used to evaluate the impact of preventive strategies and reduce the burden of infection in the suffering community. To achieve this aim, we extend the compartmental SEIR model by considering some nonpharmaceutical interventions to enable the effective and standard means of curbing the COVID-19 pandemic. To gain a more accurate view, mathematical analysis including positivity, boundedness, disease-free, and endemic equilibrium stability points is investigated for the dynamics of the model. Numerical simulations illustrate that the model fitting is in good agreement with the actual data of COVID-19-infected cases in Egypt. The basic reproduction number *ℛ*_0_, as an epidemic threshold to determine how the disease is transmitted, is calculated for the proposed model via the next-generation matrix method. We have examined the locally and globally asymptotically stable of the disease-free and endemic equilibrium points via the Routh-Hurwitz stability criterion and Lyapunov function candidate in terms of *ℛ*_0_. Accordingly, in the case of *ℛ*_0_ < 1, the disease can be eradicated. Otherwise, if *ℛ*_0_ > 1, then the disease will persist and spread in the community. The parameters used in the model simulations are estimated using the nonlinear least squares approach for the best fit between the reported cumulative data of COVID-19 from 14 February to 23 May, 2020, in Egypt and the solution of the proposed model. Based on the obtained numerical values of the model parameters, the estimated value of *ℛ*_0_ is 2.6408, which includes the effects of different infected compartments as *ℛ*_*I*_*a*__ ≈ 1.4292, *ℛ*_*I*_*s*__ ≈ 1.1855, and *ℛ*_*Q*_ ≈ 0.0261.

The impact of some model parameters that are considered preventive interventions in order to meet the flattening curve for COVID-19 is examined. Based on our findings, three nonpharmaceutical prevention measures, including increasing the physical distance to reduce the contact rate, performing the contact-tracing process, and imposing compulsory quarantine on exposed individuals, are the most influential policies and play an effective role in improving the idea of fitting curves in society and reducing treatment costs substantially. The sensitivity analysis revealed that rigorous compliance with social distancing regulations (at least a 40% decrease in *β* compared to its baseline value) is the most effective parameter in mitigating disease spread, followed by *ε*_1_ and the quarantine rate for exposed individuals, denoted by *ν*. In addition, the effect of changes in a pair of model parameters simultaneously on the numerical value of *ℛ*_0_ has been depicted. The results confirm that in the absence of pharmacological measures such as vaccine allocation and administration, strict physical distancing, self-isolation intervention, and improvement of the quality of medical infrastructure in order to reduce the peak number of infected people are a priority.

However, due to the deficiency of basic infrastructure in developing countries such as Egypt, the rigorous implementation of preventive protocols simultaneously is always challenging for the government. Therefore, by rigorous implementation of social distancing measures, proper monitoring of exposed people, and self-quarantine at home, the burden of the disease can be tackled on the suffering community. In future work, we will enhance the proposed model by introducing the effect of vaccination allocation and designing the time-dependent optimal control strategy as effective treatment measures. In this case, the effects of the basic nonpharmaceutical protocols (constant control) and therapeutic measures (optimal control) will be examined, and the results will be compared.

## Figures and Tables

**Figure 1:** Compartmental flow diagram of COVID-19 transmission in Egypt, where *λ* = *β*(*I*_*s*_ + *ε*_1_*I*_*a*_ + *ε*_2_*Q*)/*N*.

**Figure 2:** Model fitting to the cumulative reported cases from 14 February to 23 May 2020 in Egypt.

**Figure 3:** Comparison and prediction of cumulative symptomatic infectious cases with real data (red circles) in Egypt until Sep 1, 2020.

**Figure 4:** Sensitivity indices of COVID-19 model.

**Figure 5:** Effect of contact rate *β* on the variation of confirmed COVID-19 cases in Egypt.

**Figure 6:** Effect of transmission rate (*ε*_1_) from asymptomatic individuals on the variation of confirmed COVID-19 cases in Egypt.

**Figure 7:** Effect of transmission rate (*ε*_2_) related to quarantine/self-isolation individuals on the variation of confirmed COVID-19 cases in Egypt.

**Figure 8:** Effect of increasing the quarantine rate (*ν*) of exposed individuals on the variation of confirmed COVID-19 cases in Egypt.

**Figure 9:** Effect of increasing hospitalization rate of symptomatic individuals (*δ*) on the variation of confirmed COVID-19 cases in Egypt.

**Figure 10:** The behavior of the basic reproduction number (a) surface plot and (b) contour plot, in terms of *ε*_1_ and *ε*_2_. Given that, the rest of the parameters are fixed and are taken from Table 3. The color bar represents the numerical value of *ℛ*_0_.

**Figure 11:** The behavior of the basic reproduction number (a) surface plot and (b) contour plot, in terms of *δ* and *φ*. Given that, the rest of the parameters are fixed and are taken from Table 3. The color bar represents the numerical value of *ℛ*_0_.

**Figure 12:** The behavior of the basic reproduction number (a) surface plot and (b) contour plot, in terms of *ν* and *β*. Given that, the rest of the parameters are fixed and are taken from Table 3. The color bar represents the numerical value of *ℛ*_0_.

**Figure 13:** The behavior of the basic reproduction number (a) surface plot and (b) contour plot, in terms of *β* and *δ*. Given that, the rest of the parameters are fixed and are taken from Table 3. The color bar represents the numerical value of *ℛ*_0_.

**Figure 14:** Dynamical behavior of model trajectories corresponding to (a) asymptomatic individuals, (b) symptomatic individuals, and (c) exposed individuals at different initial conditions, according to Theorem 4. For this purpose, all parameters are taken from Table 3, except *β* = 0.19416 and *δ* = 0.02035; therefore, *ℛ*_0_ = 0.7860 < 1.

**Table 1:** Interpretation of the COVID-19 model parameters.

Parameters	Biological description
*N*	Total human population size
*μ*_*d*_	Per capita death rate (inverse of life expectancy)
*Π*	Recruitment rate of people
*ε*_1_	Effective transmission rate of infection from asymptomatic individuals
*ε*_2_	Proportion of quarantine effect on effective contact rate
*φ* ^−1^	Incubation period of coronavirus
*ς*	Proportion of asymptomatically infected cases after the incubation period
*σ*	COVID-19-induced mortality rate in *I*_*s*_ class
*δ*	Hospitalization rate of symptomatic individuals
*r*	Recovery rate from quarantined individuals
*α*	Rate of recovery for asymptomatic individuals
*θ*	Recovery rate from symptomatic individuals
*h*	Rate of recovery for hospitalized patients
*ν*	Quarantine rate of exposed individuals
*β*	Virus transmission coefficient
*q*	Rate of hospitalization from quarantined infected populations
*w*	COVID-19-induced mortality rate in *Q* class
*ξ*	COVID-19-induced death rate in *H* class

**Table 2:** Sign of sensitivity indices for *ℛ*_0._

Notation	Sensitivity indices
*ε*_1_	+ve
*ε*_2_	+ve
*β*	+ve
*ς*	+ve
*φ*	-ve
*δ*	-ve
*α*	-ve
*θ*	-ve
*ν*	-ve

**Table 3:** Values of biological parameters used in simulations of the COVID-19 model in Egypt 2020.

Parameters	Biological interpretation	Value (unit)	Reference
*N*(0)	Total human population size	102,334,404 (individual)	[32]
*μ*_*d*_	Per capita death rate (inverse of life expectancy)	1/72.54 × 365 (1/day)	[32]
*Π*	Recruitment rate of people	*N* × *μ*_*d*_ (1/day)	Estimated
*σ*	COVID-19-induced mortality rate in *I*_*s*_ class	0.05801 (1/day)	Fitted
*ε*_1_	Effective transmission rate of infection from asymptomatic individuals	0.13980	Fitted
*ε*_2_	Proportion of quarantine effect on effective contact rate	0.10941	Fitted
*δ*	Hospitalization rate of symptomatic individuals	2.814 × 10^−5^ (1/day)	Fitted
*ς*	Proportion of asymptomatically infected cases after the incubation period	0.30078	Fitted
*φ* ^−1^	Average incubation period of coronavirus	1/0.14285 (day)	Fitted
*r*	Recovery rate from quarantined individuals	0.80338 (1/day)	Fitted
*α*	Rate of recovery for asymptomatic individuals	9.54 × 10^−3^ (1/day)	Fitted
*θ*	Recovery rate from symptomatic individuals	0.14285 (1/day)	Fitted
*h*	Rate of recovery for hospitalized patients	0.49839 (1/day)	Fitted
*ν*	Quarantine rate of exposed individuals	0.13134 (1/day)	Fitted
*β*	Virus transmission coefficient	0.65317 (1/day)	Fitted
*q*	Rate of hospitalization from quarantined infected populations	0.44649 (1/day)	Fitted
*w*	COVID-19-induced mortality rate in *Q* class	0.05781 (1/day)	Fitted
*ξ*	COVID-19-induced death rate in *H* class	0.05801 (1/day)	Fitted

## Data Availability

No data were used to support this study.
